# Communication of Autonomous Vehicles in Road Accidents for Emergency Help in Healthcare Industries

**DOI:** 10.1155/2022/2506830

**Published:** 2022-01-25

**Authors:** D. Prem Raja, V. Vasudevan

**Affiliations:** Department of Information Technology, Kalasalingam Academy of Research and Education, Virudhunagar, India

## Abstract

Autonomous cars like driverless motors are considered solely in science fiction films; however, in 2019, they are turning into a veracity and reality. People all around the world are excited to see the driverless automobile in reality. Selfless vehicles do not want human intervention. A completely driverless car is nonetheless at a superior trying out stage; however, in part due to computerized technological know-how, it has been around for the last few years. A partly computerized car has points such as lane keeping, automatic braking, and adaptive cruise control. With a self-sustaining automobile device, the vehicle has to feel the environment and discover objects, and with the assistance of GPS, it should run on the right navigation course even while obeying site visitors and transportation rules. In addition to that, the safety of passengers and pedestrians is also very important. This capability to keep away from collisions with barriers and accidents during assemble is important. To forestall the self-sufficient vehicle, this autonomous system helps a lot. The sensor used in this gadget identifies the objects in front of the car and stops the car, directing it to go on a specific course to keep away from accidents and communicate with each other. This accident-avoidance gadget and communication system help the self-sustaining car to attain the vacation spot via coaching the vehicle with synthetic intelligence. By making the motors smartest the lifestyles fashion additionally turns into smartest.

## 1. Introduction

Driving is an obligatory exercise for most people. People use their vehicles to pass from one region to different place. The wide variety of cars available is growing day by day. It is produced in a tightly tacked manner and is prone to accidents. Nowadays, the number of accidents is so excessive and uncertain. Accidents occur each and every time, in all places and for all reasons, resulting in the worst damage, serious harm, and death. Accidents are prompted, in the main, due to the lengthening use of brakes. This work is designed to boost a new device that can resolve this hassle the place drivers might also now not brake manually however the cars can end mechanically due to obstacles [1]. This work is about a machine that can manage braking devices for safety. Using ultrasonic as a ranging sensor, its characteristics are based totally on ultrasonic waves. After transmitting by using a transmitter, the wave can mirror when an impediment is detected and gotten hold of by using a receiver. The primary goal for this mission is a self-reliant auto that can brake due to boundaries when the sensor senses the obstacles. The braking circuit function is to brake the auto mechanically after obtaining a sign from the sensor. To forestall these accidents of automobiles from taking place, we are utilizing ultrasonic sensors [2].

Loss of lives due to an ambulance stuck in traffic can be avoided by incorporating a special system in self-driving vehicles which will move aside the vehicles and let the ambulance pass by. A camera is fixed on the back of the car taking a line feed of the surroundings. From the feed, frames are fed to the deep learning module which detects ambulances from the frames. The technology used in the detection of ambulances from frames of the live feed is the convolutional neutral network. The ambulance can just be communicating and need not be in an emergency state always, so no need to provide way to ambulance is their situations. To implement the recognition of an emergency state or not, an audio detection module is used. The audio from the surroundings is taken through a microphone and an audio duration of 10 seconds is fed to the sound detection module, which uses support vector machine, normally known as SVM and gives out the output of whether there is an ambulance in the surrounding or not. Based on the results of both the modules, i.e., image detection and audio detection, an ambulance is detected in the surrounding area and proper action is taken.

There are numerous advanced science and improvements available for automobile safety. Even though there are superior technological improvements for automobile safety, the range of accidents is constantly increasing [3]. And these accidents are due to collisions or intersectional accidents. Collisions of cars take place due to errors made by the driver and intersectional accidents are brought about due to horrific climate conditions [4]. Hence, to overcome these errors, a clever collision avoidance gadget is proposed. So, the errors achieved by using the driver are eliminated. Only sports activity motors and different luxurious motors consist of antilock brake systems, velocity sensors, and different computerized systems. But these automobiles cannot be less expensive to everyone. So, this gadget has been developed which can be applied in each car [5]. A collision avoidance machine consists of numerous sensors that are installed inside an automobile which furnish warnings to the driver if there are any risks that lie ahead on the road. These sensors encompass how close the vehicle is to different cars, how much its velocity wants to be decreased when barriers are nearer to the car, and how close the auto is to going off the road [6]. The gadget consists of an audio warning to alert the driver that initiates braking if the driver fails to reply to the warning. The machine consists of sensors which ship and get hold of indicators from different cars and barriers on the road. A proper instance of the device is how it works when a driver is about to exchange lanes and there is an impediment in his blind spot [7]. The sensor will realize that impediment and provide facts to the driver before he begins turning his car and forestall him from getting into a serious accident [8]. There are a lot of strategies accessible for distance measurements and to keep away from collisions in advance; however, the one approach which is implemented in our machine and is fast, effective, and lower priced is by using ultrasonic sensors. An ultrasonic sensor is used to measure the distance with appreciation to the previous car [9]. Hence, the rear-end collision can be averted by using ultrasonic sensor. This research work effectively avoids accidents in a significant manner by applying the brake properly at a right situation in the right direction.

The paper has been organized as follows: Section 2 discusses related works, Section 3 discusses about the proposed research work, Sections 4 and 5 discuss algorithm and communication protocols. Finally, Section 6 concludes the article.

## 2. Related Work

### 2.1. Road Accident Rates

In India, 130,000 deaths occur per year. With this record, India overhauled China with the very bad rate of road accidents in the world. As per the record, 1, 39, 091 people lost their lives in 4, 40, 042 road accidents in the nation the previous year. The data given by the National Crime Records Bureau (NCRB) shows that 1, 18, 533 of the fatalities were males which includes 11,571 pedestrians. The remaining 1, 36, 771 deaths happened in all over 28 states and the seven Union Territories. Tamil Nadu is at the top of the list with 16,175 deaths in 67,757 accidents [10]. Based on the road accident report for 2014 prepared by the road transport and highway ministry, 75,000 individuals have been killed because of the killer roads of India (Figure 1).

Since India is a developing country, we are focusing on our infrastructure development and digitalizing the country with the help of technology. Related to that, India is also working on the automobile industry to build a successful autonomous vehicle which drives on its own without the help of any human. Autonomous vehicles are becoming a reality all over the world by 2020. Now a days some of the cars are developed with an advanced detection of accident system (ADAS) in which, if the vehicle finds any vehicle or pedestrian in front of it, the alert signal is given to the driver and there is declining in speed and the activation of antibraking system. This is not much efficient and causes accidents in some cases [11]. Causes of road accidents are illustrated in Figure 2. This ADAS is not able to work properly because of bad weather and low light density conditions and leads to obstacle collisions. The automation is becoming a buzz and a bliss word in each and every field. In the automobile industry, the autonomous vehicles are becoming a new evolving technology the world waits for.

Even though the automated machines reduce our work and manpower, it is difficult to trust the machine blindly when it comes to safety and security. As a human, making errors is natural, even though it may lead to the loss of life, but the chances are also a little less than the automated machines [12].

### 2.2. Autonomous Car Accident Cases

Self-driving cars initially appeared on public roadways in the year 2013. Since it started, the major focus of the manufactures has been to build an autonomous vehicle that is safe, preventive, with good logical thinking and decision making that is safer than a human controlled car [13]. Autonomous vehicles have various advantages, from harmless driving behaviors to a smaller amount of jamming in the cities and towns. Selfless driving car will not mean the termination of road traffic accidents. Obstacle collisions can happen as the outcome of both human's fault and technical mistake [14].

Research nowadays predicts that by 2050, proudly owning a clever self-reliant car will grow to be the norm for consumers [15]. The first large bounce in introducing independent cars to the client market is predicted in 2017 by Google, whose self-driving technological know-how now charges a tenth of its unique $80,000 rate tag. Every foremost automobile producer will probably comply with the aid of the early 2020s [16]. Many of the key portions of technological know-how essential for the manufacturing of self-reliant motors are persevering with a reduction in value as the technological know-how is perfected. And whilst the fee of a self-driving automobile is still in the backyard, the charge varies for most consumers, and investor interest continues to increase [17].

According to a University of Texas report, if ninety per cent of the automobiles on roads in the United States have been replaced by independent vehicles, the financial savings across a variety of industries, such as automakers, insurers, and the government, ought to attain as high as $450 billion [18]. This would be a large incentive for policymakers to clear the way for self-driving motors in the future. The full adoption of self-sufficient cars will possibly take decades, but the anticipated safety, economic system, and comfort will no doubt assist in pacing up the process [19].  Figure 3 shows the countries which are stepping towards autonomous vehicles.

## 3. Proposed Work

The idea is to stop the accident with the useful resource of calculating the distance. Many different sciences were used to avoid the accident, but none of them used ultrasonic. The boundaries of exceptional utilized sciences have been reduced to an incredible extent. An approach to stopping an accident through the utilization of science is referred to as ultrasonic. This task focuses on developing an easy laptop that specializes in detecting intrusions and doing shut differ obstacle detection. Automobile safety can be accelerated by way of the ability of looking forward to a crash earlier than it takes place, thereby imparting more time to set up protection technologies. Warnings can be like buzzers. If the driver is drawing close to a pothole or any obstruction, the driver would possibly be warned in the best way possible involving what the avenue entails. The research work's ultimate reason was consequently finalized as being one to assemble a general, easy-to-use, and versatile gadget that can give up lethal accidents. Many technological boundaries in the cutting-edge computer have been attempted to be overcome in our proposed system. Our proposed machine is about stopping lethal accidents through the utilization of ultrasonics. Our essential intention is to calculate the distance between the car and an obstacle. It is shown in Figure 4.

The module used is HC-SR04 ranging from 50 cm. The sensor consists of an ultrasonic transmitter, a receiver, and a manage circuit. It consists of four pins: VCC of 5 v, enter set off pulse, output echo pulse, and ground. The electric powered parameter of ultrasonic sensor are as follows: its working voltage is 5 v DC; its working frequency is forty kHz. It has prompted enter sign of 10 us TTL pulse. An ultrasonic sensor works on the simple precept of piezoelectric effect. To set off, a quick 10 us pulse is supplied, and then the module will ship an eight-cycle sonic burst of ultrasound having a frequency of forty kHz. Once the impediment is detected, the mirrored waves (echo) are sensed by the receiver and analyzed by the microcontroller. If the distance is not in the protected limit, then the microcontroller will display a warning sign to the driver. When the acquired echo is dwindled away, the subsequent set off pulse is dispatched, and this time duration is known as the cycle period. The HC-SR04 cycle length has to be no longer under 50 ms.

An ambulance tacking system (ATS) is the need of the hour due to the recent pandemic situation going on around us. It is necessary that patient-caring vehicles such as ambulances must be equipped with the ATS technology. The ATS technology helps the hospital administration carry out the necessary steps before the patient arrives at the hospital premises.

### 3.1. Servo Motor

Servo means feedback. So a servo is an actuator that takes remarks itself and strikes precisely. An example of preciseness and remarks can be understood from an everyday existence example, when you pull up/down the glass of your vehicle window, you push up/down the electrical window button and stare at the actual attribute of the glass, as it reaches the desired attribute, you release the button. So this is feedback, we are taking remarks here, if it were a completely primarily based on laptop, we would have to inform the open window of 10%–20%. Servo refers to an error-sensing remarks manipulation which is used to improve the ordinary, typical overall performance of a system. Servo or RC servo motors are DC motors geared up with a servo mechanism for specific manipulation of angular position. The RC servo motors typically have a rotation restrict from 90° to 180°. In addition, some servos have a rotation limit of 360° or more. But servos do no longer rotate continually. Their rotation is restrained in between the steady angles.

### 3.2. Uses of Servo Motor

The servo motors are used for precision positioning. They are used in robotic palms and legs, sensor scanners, and in RC toys like RC helicopters, airplanes, and cars. The servo motor rotates from zero diploma to 180 degrees. We ship the command to servo, and as it reaches the commanded price, it stops there.

### 3.3. Servo and Arduino

The Arduino has received a library to control servo. It is–Servo.h. This library can manipulate the abovementioned validated servo motors. This library helps up to 12 servos on most Arduino boards and forty-eight servos on the Arduino Mega. It disables analogWrite() for Pin 9 and Pin 10 without Arduino Mega. It is illustrated in Figure 5.

### 3.4. Servo Motor Control

The servo motor can be moved to a favored angular function by means of sending PWM (pulse width modulated) indicators on the manipulate wire. The servo is familiar with the DC motor.

The DC motor is the most commonly used actuator for producing continuous movement and whose tempo of rotation can without difficulty be controlled, making them nice for use in functions such as pace control, servo form control, and/or positioning is required. A DC motor consists of two parts: a “Stator” which is the stationary section, and a “Rotor” which is the rotating part.

## 4. Techniques Involved

Rather than building a driverless car, it is also much more important to prevent that car or vehicle from accidents. It is a major factor. To achieve this, there are some techniques.

### 4.1. Real-Time Path Optimization

While driving, the driverless vehicle selects the path or route to reach its destination with the help of navigation and GPS to find the best route. While traveling, the autonomous vehicles comes in contact with the other vehicles on the road and the traffic management infrastructure to fit in with real-time information on road conditions and traffic echelons into path selection.

The increase in protection for passengers inside the vehicle and pedestrians on the road will be another prior value. The proposed accident avoidance system (AAS) in autonomous vehicles takes the challenging factor out of the driverless vehicle and will not subsidize to enhance traffic management but also increase safety, protecting human lives by reducing accidents.

### 4.2. Driven by Technology

In driverless vehicles, some of the precarious technologies behind safe and well-organized autonomous vehicle performance are artificial intelligence, machine learning, safety and security, cameras, sensor technologies radar, ultrasonic sensors and LiDAR, and sensor node network infrastructure. Every technology is integrated without a glitch to provide and ensure preventive and successful autonomous vehicle performance.

### 4.3. Artificial Intelligence

Many innovative ideas are followed in autonomous vehicles for testing and building the driverless car with the combination of various technologies. With the help of various sensors, the automated vehicle performs several tasks such as speech and voice recognition, image recognition and processing, motion detection, and data analysis which are basically neuronal activities. After integration of those functions, this helps the car to identify pedestrian motions, traffic, and other vehicles on the road, as well as traffic signals and sign boards, and follow the mapped route.

### 4.4. Safety and Security

The acceptance of autonomous vehicle is possible when there is an assurance of safety and security for the passengers and pedestrians. This accident avoidance system ensures everyone's safety and also the machine's safety. This safety is ensured because of the training given to the vehicle, as machine learning and neural thinking as well as logical thinking.

For consistent safety, the vehicles are equipped with many cameras and different kinds of sensors to observe the peripheral environment carefully where the vehicle is operating. When the infrastructure of the road and the vehicles grows and more develops, more sensors will be included to provide safe operations in autonomous vehicles.

### 4.5. Network Infrastructure

Prompt and reliable connectivity between driverless vehicles and external sources such as cloud management confirms signals received to and from the vehicles in a speedy manner.

## 5. Communication

An autonomous vehicle communicates to the peripheral environment with the help of different algorithms and protocols. This is stated as V2X or vehicles to everything is as follows:

- Vehicle to infrastructure communication: The autonomous vehicle communicates with the external atmosphere and exchanges data to perform within the constraints of speed limits, traffic lights, and signals. It helps to conserve fuel as well as the economy and avoid accidents or obstacle collisions [20].
- Vehicle to vehicle communication: When the autonomous vehicle comes into contact with other vehicles, it performs an action to prevent collisions and manage traffic situations with the help of many sensors and technologies embedded in it [20].

GSM and GPS are used for efficient working of this device. In this system, a low-cost microcontroller-based electronic device, the Arduino is used to control the GPS and GSM modules. In this system, modern display devices such as liquid crystal displays (LCDs) are used at the user end which is also called as the base station. Information regarding the location of the ambulance is provided by the GPS module. The GSM module is used for communication with the base station. The hospital administration can get information of the arrival of the ambulance well in time and can increase the chance of survival of the patient as the time required for setting up basic components is done well in advance. This system can also be used for various other vehicles used in emergency situations.

## 6. Algorithm

### 6.1. Sensor Technology

Without sensors and sensor technology, meeting the expectations of autonomous vehicles is challenging. To encounter the challenges and ensure the vehicle's operation, we use ultrasonic sensors, infrared sensors, radar, etc. These technologies enhance the vehicles in various stages.

  Stage 1: initially, to avoid accidents, the vehicle performs tasks such as controlling the steering or acceleration and maintaining a low speed
  Stage 2: in this stage, the vehicle gets alerted about the obstacle and recognizes it
  Stage 3: the vehicle performs “safety-critical functions” from various traffic and external sources, surroundings, and conditions
  Stage 4: the vehicle reacts according to the obstacle, which is either static or dynamic (object in motion)
  Stage 5: vehicles work with full automation by giving signals either as text or speech in any environment with the help of proper navigation

It is shown in Figure 6. Block diagram is illustrated in Figure 7.

## 7. Conclusion and Future Work

The proposed machine is designed into a small automobile mannequin as a prototype to manage the distance between the automobile and the preceding automobile, and additionally, the distance between the front boundaries and initiate automated braking. A rear-end accident avoidance device is designed and hooked up on a very easy and without difficulty comprehensible mannequin developed to show the device and its use. It was discovered to be functional. The sensor was once in a position to study distances that are short and vary accurately.

A distance sensor that detects objects at lengthy distances is required to practice on an actual vehicle. Therefore, if the proper substances are collected, it is feasible to decorate its points so that it can be used in vehicles. This mannequin is additionally a desirable device to use for demonstration of anticollision warning machine research. This device is used in thoroughly automated automobiles with adaptive cruise control. The average protection will be enhanced in addition.

Advanced driver assistant structures and new sensing applied sciences can be particularly beneficial, along with a massive physique of work on computerized vehicles. These findings advocate that the lookup into self-reliant automobiles inside the ITS area is a quick time period actuality and a promising lookup region, and these outcomes represent the beginning factor for future developments.

## Figures and Tables

**Figure 1:** Accident statistics in major cities of India [11].

**Figure 2:** Causes for road accidents.

**Figure 3:** Countries stepping towards AVs.

**Figure 4:** Ultrasonic sensor working.

**Figure 5:** Servo motor configurations.

**Figure 6:** Flow diagram for the accident avoidance system.

**Figure 7:** Block diagram for an accident avoidance system.

## Data Availability

The data supporting this research article are available from the corresponding author on reasonable request.
